The article "Detection and Functional Characterization of a 215 Amino Acid N-Terminal Extension in the Xanthomonas Type III Effector XopD" was retracted in 2018. Reasons: manipulated images; duplicated images.

# Detection and Functional Characterization of a 215 Amino Acid N-Terminal Extension in the *Xanthomonas* Type III Effector XopD

**DOI:** 10.1371/journal.pone.0015773

**Published:** 2010-12-22

**Authors:** Joanne Canonne, Daniel Marino, Laurent D. Noël, Ignacio Arechaga, Carole Pichereaux, Michel Rossignol, Dominique Roby, Susana Rivas

**Affiliations:** 1 Laboratoire des Interactions Plantes Micro-organismes (LIPM), UMR CNRS-INRA 2594/441, Castanet Tolosan, France; 2 Institut Fédératif de Recherche (IFR40), Plateforme protéomique Génopole Toulouse Midi-Pyrénées, Institut de Pharmacologie et Biologie Structurale, Université de Toulouse, Toulouse, France; 3 Departamento de Biología Molecular, Universidad de Cantabria (UC) and Instituto de Biomedicina y Biotecnología de Cantabria, IBBTEC (CSIC-UC-IDICAN), Santander, Spain; Ecole Normale Superieure, France

## Abstract

During evolution, pathogens have developed a variety of strategies to suppress plant-triggered immunity and promote successful infection. In Gram-negative phytopathogenic bacteria, the so-called type III protein secretion system works as a molecular syringe to inject type III effectors (T3Es) into plant cells. The XopD T3E from the strain 85-10 of *Xanthomonas campestris* pathovar *vesicatoria* (*Xcv*) delays the onset of symptom development and alters basal defence responses to promote pathogen growth in infected tomato leaves. XopD was previously described as a modular protein that contains (i) an N-terminal DNA-binding domain (DBD), (ii) two tandemly repeated EAR (ERF-associated amphiphillic repression) motifs involved in transcriptional repression, and (iii) a C-terminal cysteine protease domain, involved in release of SUMO (small ubiquitin-like modifier) from SUMO-modified proteins. Here, we show that the XopD protein that is produced and secreted by *Xcv* presents an additional N-terminal extension of 215 amino acids. Closer analysis of this newly identified N-terminal domain shows a low complexity region rich in lysine, alanine and glutamic acid residues (KAE-rich) with high propensity to form coiled-coil structures that confers to XopD the ability to form dimers when expressed in *E. coli*. The full length XopD protein identified in this study (XopD^1-760^) displays stronger repression of the XopD plant target promoter *PR1*, as compared to the XopD version annotated in the public databases (XopD^216-760^). Furthermore, the N-terminal extension of XopD, which is absent in XopD^216-760^, is essential for XopD type III-dependent secretion and, therefore, for complementation of an *Xcv* mutant strain deleted from XopD in its ability to delay symptom development in tomato susceptible cultivars. The identification of the complete sequence of XopD opens new perspectives for future studies on the XopD protein and its virulence-associated functions *in planta*.

The article "Detection and Functional Characterization of a 215 Amino Acid N-Terminal Extension in the Xanthomonas Type III Effector XopD" was retracted in 2018. Reasons: manipulated images; duplicated images.

## Introduction

Plants have developed a complex defence network to fight off invading pathogens. The first layer of plant defence involves recognition of PAMPs (Pathogen-Associated Molecular Patterns), defined as invariant epitopes within molecules that are fundamental to pathogen fitness and widely distributed among different microbes [1]. This recognition, previously known as basal defence, is now referred to as PAMP-triggered immunity (PTI) [2]. PTI is associated to the production of reactive oxygen species and antimicrobial compounds, the induction of mitogen-activated protein kinase (MAPK) cascades, the modulation of host gene transcription and the deposition of lignin and callose at the plant cell wall [3]–[6]. Some bacterial pathogens evolved to suppress PTI and promote successful infection by injecting T3Es (type III effectors) into plant cells using the type III protein secretion system (T3SS) [7]–[9]. In turn, plants acquired the ability to recognize directly or indirectly effectors through resistance (R) proteins. This recognition response is associated with the long-standing gene-for-gene hypothesis, and more recently with the guard hypothesis [10], and is now known as effector-triggered immunity (ETI). Several T3Es from Gram-negative phytopathogenic bacteria have also been shown to suppress ETI [11], suggesting that T3Es may have multiple targets or that they target shared components between PTI and ETI.

The coevolutionary arms race between plants and pathogens has generated highly polymorphic repertoires of R proteins and T3Es. A significant number of T3Es from different bacteria has been identified during the last few years. Known biochemical activities of T3Es include manipulation of host protein turnover, either through protease activity [12]–[14] or protein degradation via the 26S proteasome [15]–[17], modification of host transcription or RNA stability [18]–[21] and alteration of the phosphorylation state of plant proteins [22]–[27].

Gram-negative pathogenic bacteria of the genus *Xanthomonas* infect a wide range of host plants and are responsible for important crop plant diseases. *Xanthomonas campestris* pathovar *vesicatoria* (*Xcv*, also known as *Xanthomonas axonopodis* pathovar *vesicatoria* or *Xanthomonas euvesicatoria* [28], [29]) is the causal agent of bacterial spot on tomato (*Solanum lycopersicum*) and pepper (*Capsicum annum*) [30]. The T3SS of *Xcv* is encoded by the chromosomal *hrp* (HR and pathogenicity) gene cluster, which contains 25 genes [31], [32]. *hrp* gene expression is activated during plant infection or when bacteria are incubated in special minimal media by two regulatory proteins, HrpG and HrpX. HrpG is a member of the OmpR family of two-component system response regulators and controls the expression of a genome-wide regulon including *hrpX* [33], [34]. HrpX is an AraC-type transcriptional activator that binds to a conserved DNA motif [plant-inducible promoter (PIP) box; consensus: TTCGC-N15-TTCGC], which is present in the promoter regions of most *hrpX-*regulated genes [33], [35].

The article "Detection and Functional Characterization of a 215 Amino Acid N-Terminal Extension in the Xanthomonas Type III Effector XopD" was retracted in 2018. Reasons: manipulated images; duplicated images.

T3SS-dependent secretion of a protein is mediated by an N-terminal secretion signal within its first 15–20 residues. The presence of hydrophilic amino acids, absence of acidic residues in the first 12 amino acids, amphipacity and a bias towards serine and glutamine in the first 50 residues are common features of the N-terminal sequence of T3Es [36]–[39]. In addition to the secretion signal, effector proteins contain a 1–50 to 1–100 amino acid region at their N-terminus that is required for translocation across the eukaryotic plasma membrane [40].

The presence of a variety of putative structural motifs in the primary sequence of *Xanthomonas* T3Es has provided insights into their putative biochemical function [41]. The XopD T3E from *Xcv* 85-10 has been classified as a member of the C48 protease family, and it has been shown to release SUMO (small ubiquitin-like modifier) from SUMO-modified plant proteins [42], [43]. XopD is a modular protein that contains (i) an N-terminal DNA-binding domain (DBD), (ii) two tandemly repeated EAR (ERF-associated amphiphillic repression) motifs [^L^/_F_DLN^L^/_F_(X)P] [44], previously described in plant transcriptional repressors that negatively regulate gene transcription during stress and defence responses [45], and (iii) a C-terminal cysteine protease domain with structural similarity with the yeast ubiquitin-like protease 1 (ULP1) [42]. XopD is localized in nuclear foci indicating that host targets are likely nuclear SUMOylated proteins [43]. Intriguingly, consistent with its protein structure, XopD has been reported to be a non-specific DNA-binding protein that represses plant gene transcription, delaying the onset of symptom development and altering basal defence and cell death responses, which in turn promotes pathogen growth in infected leaves [46]. However, as for many of the known bacterial effectors, XopD direct plant targets remain unknown.

*XopD* was previously predicted to code for a protein of 612 amino acids [47]. However, secretion assays and Western blot analysis, following expression of c-myc-tagged XopD within its native *Xcv* chromosomic environment, allowed the detection of a unique band of a molecular mass close to 100 kDa [47]. Importantly, this protein was undetectable in culture supernatants of T3SS mutant bacteria cultured in secretion medium, demonstrating that this protein is secreted in a T3SS-dependent manner. In contrast, the XopD protein sequence annotated in the public databases predicts a protein of 545 amino acids with an expected molecular mass of 61 kDa. Noël and co-workers could not detect a (consensus) PIP box in the *xopD* promoter, but rather a putative *hrp* box, which is found in all *hrpL*-dependent promoters in *Pseudomonas syringae* and *Erwinia* spp [47]–[49]. Later inspection of the *xopD* promoter region identified the presence of a PIP box (ATCGC-N15-TTCGT), bound by HrpX, and a −10 putative sequence (TAAATT), which are situated 747 and 690 bp upstream the annotated start, respectively (Figure 1A) [35]. In agreement with these observations, the HrpX-dependent expression of XopD has been confirmed experimentally [35], [47].

The article "Detection and Functional Characterization of a 215 Amino Acid N-Terminal Extension in the Xanthomonas Type III Effector XopD" was retracted in 2018. Reasons: manipulated images; duplicated images.

**Figure 1:** *In silico* analysis of the *xopD* locus. (A) The *xopD* locus in *Xcv* 85-10 is shown (the genome interval for the *Xcv* 85-10 shown sequence and the *xopD* gene are respectively: 486209–489200 and 486544–488826). Open arrows indicate ORFs and filled arrows show promoter elements, such as the PIP box and the −10 sequence. The position of XopD translation start annotated in the public databases is indicated by an asterisk. (**B**) Schematic representation of XopD functional domains in *Xcv* 85-10, in comparison to its known protein homologues. The N-terminal extension, essential V and L residues in the DBD, tandemly repeated EAR motifs, conserved catalytic residues in the cysteine protease domain, and NLS motif are shown. (**C**) Sequence alignment of XopD from *Xcv* 85-10, hypothetical protein from *Xcc* B100 (YP_001902662), virulence protein from *Xcc* 8004 (AAY48282) or *Xcc* ATCC 33913 (AAM42168), peptidase C48 SUMO from *Acidovorax avenae* (EFA39722) and XopD from *Xcc* 147. The figure shows the longest ORF possible for all proteins. For XopD from *Xcv*, the first shown M residue corresponds to a UUG codon, not conserved among *Xcc* B100 and *A. avenae* coding sequences. The M residue previously annotated as the starting amino acid of the XopD protein is indicated by a red arrowhead. Putative translation starts situated in frame and upstream the previously annotated starting M are also indicated as follows: translation starts conserved among *Xcv* 85-10, *Xcc* B100 and *Aea* are indicated with a full red dot, otherwise, they appear indicated by an empty red dot. Yellow box: putative N-terminal extension; green box: DNA-binding domain (V and L residues in the helix-loop-helix domain essential for maximal DNA-binding [46] are indicated by an empty green dot); red boxes: tandemly-repeated EAR motifs [^L^/_F_DNL^L^/_F_(X)P] [44]; black box: SUMO protease domain (H, D and C catalytic core residues are indicated by a black empty dot); blue box: NLS. Gray and black highlighting of amino acids indicates, respectively, 70–80% and 90–100% of similarity.

The article "Detection and Functional Characterization of a 215 Amino Acid N-Terminal Extension in the Xanthomonas Type III Effector XopD" was retracted in 2018. Reasons: manipulated images; duplicated images.

In the view of these conflicting data, we set out to identify the starting amino acid of XopD and thereby determine the sequence of the XopD protein that is produced and secreted from *Xcv*. Our work confirms that the XopD protein sequence previously annotated in the databases is incomplete. We demonstrate that the functional protein expressed by *Xcv* presents a previously overlooked N-terminal extension of 215 amino acids that is essential for its T3SS-dependent secretion and virulence-associated functions in the plant cell.

## Results

### Sequence analysis of the *xopD* locus

In bacteria, the most frequently used codon for the initiation of translation is the triplet AUG, although GUG and, occasionally, UUG may also be used. The meaning of the GUG, or the rarely used UUG, codon depends on their context. When present within a gene, they provide valine (V), or leucine (L), as specified by the genetic code. However, present as first codons, they mediate the incorporation of methionine (M). Close inspection of the *Xcv* 85-10 genomic sequence neighbouring the annotated *xopD* gene shows that upstream of the annotated starting codon AUG, there are 6 AUG, 1 GUG and 5 UUG additional codons that are in frame and may potentially be used to start translation of the protein (Figure 1C). In addition, since HrpX-dependent expression of XopD was previously demonstrated, the presence of a PIP box and a −10 sequence upstream of the first putative starting codon suggested that translation of XopD may start immediately downstream these regulatory elements (Figure 1A).

BlastP analysis using the *Xcv* 85-10 XopD sequence starting at the first possible translation start (UUG, encoding or not a M residue depending on whether it is or not the translation start) identified three major hits corresponding to (i) a hypothetical, not yet characterized, protein from the strain B100 of *Xantomonas campestris* pathovar *campestris* (*Xcc*) [50], (ii) a protein from *Acidovorax avenae*, annotated as peptidase C48 SUMO/Sentrin/Ub11, and (iii) two virulence proteins that correspond to a shorter version of XopD deleted from its DBD, from the *Xcc* strains 8004 [51] and ATCC 33913 [52] (Figure 1B). In addition, sequencing of *xopD* using genomic DNA from the *Xcc* 147 strain [53] showed that this XopD protein is very similar to the one present in *Xcc* strains 8004 and ATCC 39913 (Figure 1B,C). It is noteworthy that the Met residue previously annotated as XopD starting amino acid is not conserved in *Xcc* B100 (Figure 1C; red arrow), suggesting that this may not be a starting amino acid for XopD. In contrast, the putative N-terminal extension of XopD is well conserved in both *A. avenae* and *Xcc* B100, indicating that it may be important for XopD function (Figure 1C).

The article "Detection and Functional Characterization of a 215 Amino Acid N-Terminal Extension in the Xanthomonas Type III Effector XopD" was retracted in 2018. Reasons: manipulated images; duplicated images.

### T3SS-dependent secretion of an 85 kDa XopD protein from *Xcv*

To allow detection of the XopD protein that is produced by *Xcv* from its native promoter, *Xcv* genomic DNA was tagged with an HA epitope at the 3′end of *xopD* coding sequence using a suicide vector. XopD protein expression was analyzed in strains 85*, which allows constitutive expression of all *hrp* genes [54], and 85* Δ*hrcV*, which carries a deletion in a conserved component of the T3SS [55]. Western blot analysis of bacterial total protein extracts with an anti-HA antibody did not allow detection of any band at ∼61 kDa, which is the predicted molecular mass of the annotated XopD protein (Figure 2). In contrast, a unique band of ∼85 kDa was detected (Figure 2, lane 1), strongly suggesting that (i) there is a unique start for XopD translation and that (ii) the protein that is produced by *Xcv* presents a significant extension at the N-terminus of the annotated protein. No HA-tagged protein could be detected in the untransformed strain 85* (Figure 2, lane 2).

**Figure 2:** Expression analysis of XopD. Strains 85* (XopD-HA) (1), 85* (2) and 85* Δ*hrcV* (XopD-HA) (3) were incubated in MOKA rich medium (total extract, left) or secretion medium (supernatant, right). Total protein extracts (10-fold concentrated) and TCA-precipitated filtered supernatants (200-fold concentrated) were analyzed by immunoblotting using anti-HA antibodies (upper panel) to detect the presence of XopD, or anti-GroEL antibodies (lower panel) to show that bacterial lysis had not occurred.

*hrp*-dependent secretion of XopD was next tested after incubation of bacteria in secretion medium. A single band of ∼85 kDa was detected in culture supernatants of the 85* strain (Figure 2, lane 1). XopD was not detectable in culture supernatants of T3SS mutant 85* Δ*hrcV* (Figure 2, lane 3), reflecting the presence of a functional T3SS secretion signal in the ∼85 kDa form of XopD. No protein could be detected in the supernatant fractions with an antibody against the intracellular chaperone GroEL, demonstrating that detection of proteins in the supernatant was not due to bacterial lysis (Figure 2).

Since the expected molecular mass for the longest possible ORF (UUG codon; Figure 1C) is 86 kDa, this analysis shows that the molecular mass of the XopD protein produced and secreted by *Xcv* 85* in a T3S-dependent manner is consistent with the protein starting at one of its very first putative translation starts.

The article "Detection and Functional Characterization of a 215 Amino Acid N-Terminal Extension in the Xanthomonas Type III Effector XopD" was retracted in 2018. Reasons: manipulated images; duplicated images.

### Identification of a 215 amino acid N-terminal extension in XopD using mass spectrometry

A mass spectrometry analysis was thus conducted to determine the starting amino acid of the XopD protein produced by *Xcv*. HA-tagged XopD was immunopurified from *Xcv* 85* cultures and subjected to electrophoresis. After Coomassie staining of the gel, a ∼85 kDa band corresponding to XopD was excised, digested with trypsin and analyzed by mass spectrometry (Nano LC/ESI MS/MS). Trypsin cleaves at the C-terminal side of arginine (R) and lysine (K) residues, which are well distributed throughout the XopD sequence. In total, 28 peptides corresponding to XopD were detected (Figure 3A; Table 1), which represents a total XopD sequence coverage of 44%. The N-terminal region of the protein was particularly well covered (58% coverage for the newly identified N-terminal extension). MS/MS fragmentations for all peptides are provided in Figure S1.

**Figure 3:** Analysis of the XopD protein sequence by mass spectrometry. XopD^216-760^ protein sequence is shadowed. All possible translation starts situated in frame and upstream the annotated M^216^ are underlined. Peptides identified by Nano LC/ESI MS/MS analysis following trypsin (A) or V8 protease (B) digestion of the purified XopD protein are shown in bold. The 30 amino acid low complexity KAE-rich region is indicated in red.

**Table 1:** Sequences and individual MASCOT scores of XopD peptides identified by Nano LC/ESI MS/MS analysis after trypsin digestion.

Peptide sequence^a^^,^ b	MASCOT score
IFNFDYK	35
EMTEAADDYR	69
ENHGAGYNMHPLLESLPR	38
RNPTQVHADGSVHQMR	60
ILELISAYGDGK	107
GIPELQR	24
QMLQELNEDQR	68
DQVIHQIIR	50
RIEYCADPEYR	34
EVALSR	25
ITLSQR	29
AKAEAEAEAK	21
INEIMEYIPR	77
YEALEK	22
GDGSFGPGLPGILR	52
YMTPDQK	20
LYLASER	28
KLALAAPK	53
TLHQKPNLLLEISSK	26
LGEAVISGASQGIQTAIR	117
AWPAQPEASSSTFDDLESLDYR	90
IDVDNLPSPQDVADPELPPVR	80
ATSWLLDGHLR	64
AYTDDLAR	49
NKDAVAAYHYDSMAQK	24
VLDGTFDYAGGR	77
DLTDIEPDR	22
LAQAEQAPAESSIR	82

a The first 13 peptides are present in the XopD N-terminal extension.

b The starting M residue for the XopD protein annotated in the public databases in underlined in the INEIMEYIPR peptide.

Detection of a peptide (INEIMEYIPR; Figure 3; Table 1) encompassing the annotated starting M^216^ residue demonstrates that the XopD sequence annotated in the public databases is not complete. Furthermore, the first detected peptide is IFNFDYK, showing that the two possible start residues for XopD are the first and the second M shown in Figures 1C and 3.

The article "Detection and Functional Characterization of a 215 Amino Acid N-Terminal Extension in the Xanthomonas Type III Effector XopD" was retracted in 2018. Reasons: manipulated images; duplicated images.

To determine the starting amino acid of XopD, we next used the V8 protease, which cleaves at the C-terminal side of glutamic (E) and aspartic acid (D) residues, before conducting the mass spectrometry analysis. In total, 15 peptides were detected, which represents a XopD sequence coverage of 21% (Figure 3B; Table 2; Figure S2). Importantly, detection of the peptide MDRIFNFD demonstrates that the XopD protein that is produced by *Xcv* starts at the second predicted M of the longest possible ORF (XopD^1-760^, Figure 1C and 3). This represents an N-terminal extension of 215 amino acids compared to the annotated XopD protein (XopD^216-760^) and conservation of this sequence in both *Xcc* B100 and *A. avenae* (Figure 1C) suggests that this region may be important for XopD function(s).

**Table 2:** Sequences and individual MASCOT scores of XopD peptides identified by Nano LC/ESI MS/MS analysis after digestion with the V8 protease.

Peptide sequence^a^ ^,b^	MASCOT score
MDRIFNFD	25
YKKYREMTE	20
NHGAGYNMHPLLE	25
LQRSFPSFAAFLMD	41
YCADPEYRE	28
VALSRLE	37
SDCSGKITLSQRTLD	49
YIPRYE	22
LTRLGE	30
SLDYRQNYGYRE	22
LPPVRATSWLLD	26
AVAAYHYD	30
SMAQKDPQQRYLAD	23
MAAYHLGLDYQQTHE	29
VLAHRVLD	39

a The first 8 peptides are present in the XopD N-terminal extension.

### XopD^1-760^ is able to form dimers in *E. coli*

To gain insight into the putative function of XopD N-terminal extension, XopD amino acid sequence (full length XopD^1-760^) was analyzed for its biochemical properties. Interestingly, we found a region rich in lysine, alanine and glutamic residues (KAE-rich; residues 168–202) with high propensity to form coiled-coil structures (Figure 4A). The presence of this type of coiled-coil structures generally indicates that the protein may interact with other amino acid chains of the same polypeptide to form oligomers or other polypeptides to form complexes. Further analysis predicted that this coiled-coil, KAE-rich region is likely to be involved in dimer formation, rather than trimer or other oligomeric structures (Figure 4A).

**Figure 4:** XopD^1-760^, but not XopD^216-760^, is able to dimerize. (**A**) Multicoil (http://groups.csail.mit.edu/cb/multicoil/cgi-bin/multicoil.cgi) prediction on XopD^1-760^ sequence. XopD amino acid sequence (amino acids 1 to 760) was analyzed for its propensity to form coiled-coil structures. A region comprising amino acid residues 168–202 showed high probability to form such coiled-coil structures. Furthermore, this coiled-coil region is likely to be involved in dimer formation (blue line), rather than trimer (red line) or other oligomeric structures. The (abcdefg) positions of the hepta-repeat in the coiled-coil region are indicated above the amino acid sequence. Above it, the relative positions of the hepta-repeat in the opposite chain within the putative dimer are indicated in blue. (**B**) Gel filtration analysis of HA-tagged XopD expressed in *Xcv*, and XopD^1-760^ and XopD^216-760^ expressed in *E. coli* as 6xHis-tagged fusions. Protein extracts were subjected to gel filtration chromatography on a Superdex S-200 column. 0.4 ml fractions were collected and aliquots were analyzed by Western blot. Fraction numbers of the elution profile re indicated by the numbers between the gels. The molecular mass estimated for each fraction (in kDa) is given at the top.

The article "Detection and Functional Characterization of a 215 Amino Acid N-Terminal Extension in the Xanthomonas Type III Effector XopD" was retracted in 2018. Reasons: manipulated images; duplicated images.

In the view of these observations, we first tested the oligomerization state of HA-tagged XopD produced by *Xcv* 85*. Size exclusion chromatography of bacterial total protein extracts, followed by Western blot analysis of the collected fractions, showed that the peak of elution of HA-tagged XopD corresponds to an estimated molecular mass of approximately 86 kDa, which coincides with the predicted molecular mass of an HA-tagged XopD monomer. This result (i) suggests that, despite the presence of a predicted coiled-coil structure, XopD is not able to dimerize in *Xcv* 85* and (ii) is consistent with the idea that, before translocation into the plant cell, T3Es are unfolded or associated to T3S chaperones to facilitate their passage through the secretion apparatus [56], [57].

The oligomerization state of XopD^1-760^ and XopD^216-760^ was next studied following overexpression of His-tagged protein versions in *E. coli* cells. The expected molecular mass for His-tagged XopD^1-760^ and XopD^216-760^ monomers is 89 and 65 kDa, respectively. After protein chromatography, aliquots from collected fractions were analyzed for the presence of XopD by immunoblot analysis. The estimated molecular mass of XopD^216-760^ ranged between 46 and 70 kDa whereas XopD^1-760^ elution ranged between 128 and 190 kDa (Figure 4B). These results strongly suggest that, consistent with the presence of a predicted coiled-coil structure, XopD^1-760^, but not XopD^216-760^, is able to dimerize in *E. coli*.

### Subcellular localization and functions of XopD^1-760^ in *N. benthamiana*

The N-terminal domain of XopD^216-760^ was previously shown to be required for targeting the effector to subnuclear foci [43]. To determine the effect of the newly identified N-terminal extension of XopD on its subcellular localization *in planta*, XopD^1-760^ was fused to the Yellow Fluorescent Protein venus (YFPv) and transiently expressed, under the control of the 35S promoter, in *Nicotiana benthamiana* leaf epidermal cells. As XopD^216-760^, XopD^1-760^ was also localized in subnuclear foci (Figure 5A). Both proteins were detected by Western blot using an anti-GFP antibody (Figure 5B).

The article "Detection and Functional Characterization of a 215 Amino Acid N-Terminal Extension in the Xanthomonas Type III Effector XopD" was retracted in 2018. Reasons: manipulated images; duplicated images.

**Figure 5:** Characterization of XopD^1-760^ expression and function in *N. benthamiana*. (**A**) Confocal images of epidermal cells of *N. benthamiana* leaves expressing YFPv-tagged XopD^216-760^ and XopD^1-760^ 36 hours after agroinfiltration. Bright field images are shown on the right. Bars  = 15 µm. (**B**) Western blot analysis using an anti-GFP antibody shows expression of YFPv-tagged XopD^216-760^ and XopD^1-760^ constructs, 36 hours after agroinfiltration. Ponceau S staining of the membrane illustrates equal loading. (**C**) Cell death development 4 (upper panel) and 7 (lower panel) days after agroinfiltration of YFPv-tagged XopD^216-760^ (left) and XopD^1-760^ (right) constructs. (**D**) Cell death was quantified by measuring electrolyte leakage in *N. benthamiana* leaves expressing YFPv-tagged XopD^216-760^ (open circles) and XopD^1-760^ (filled circles) at the indicated time points after agroinfiltration. Mean and SEM values are calculated from 3 independent experiments (8 replicates/experiment). The statistical significance in mean conductivity values obtained with leaves expressing XopD^216-760^ or XopD^1-760^ was assessed by using a Student's t test (P value <10^−5^). (**E**) SUMO-conjugates detected by Western blot analysis using an anti-HA antibody 36 hours after agroinfiltration of the indicated constructs. Expression of XopD proteins was revealed using an anti-GFP antibody. Ponceau S staining of the membrane illustrates equal loading.

*Agrobacterium*-mediated transient expression of XopD^216-760^ in *N. benthamiana* leaves results in tissue necrosis by 4 to 7 days after agroinfiltration, likely reflecting cell death due to XopD accumulation and cytotoxicity (Figure 5C; [46]). Interestingly, up to 5 days after agroinfiltration, *N. benthamiana* leaves expressing XopD^1-760^ showed a significant delay in the development of the necrotic phenotype observed after transient expression of XopD^216-760^ (Figure 5C), despite similar levels of protein accumulation (Figure 5B). These results were confirmed by ion leakage measurements in leaf disk assays, which showed significantly lower conductivity values in leaves expressing YFP-tagged XopD^1-760^, compared to leaves that expressed XopD^216-760^ (Figure 5D). These observations indicate that the N-terminal extension of XopD may negatively regulate the previously described cytotoxic effect induced by XopD^216-760^ expression. From 7 days after agroinfiltration, a similar cell death phenotype was observed with both YFP-tagged XopD^216-760^ and XopD^1-760^ (Figure 5C).

The article "Detection and Functional Characterization of a 215 Amino Acid N-Terminal Extension in the Xanthomonas Type III Effector XopD" was retracted in 2018. Reasons: manipulated images; duplicated images.

Finally, the SUMO protease activity of YFP-tagged XopD^1-760^ was investigated after co-expression with an HA-tagged *Le*SUMO construct [43] in *N. benthamiana* leaves. Western blot analysis of HA-SUMO conjugates showed that, as in the case of XopD^216-760^, expression of XopD^1-760^ led to significant reduction in the detection of SUMO-modified proteins (Figure 5E). As previously described, XopD^216-760^-C470A, mutated in the conserved Cys residue in XopD catalytic core, was not able to hydrolyze the SUMO substrates [43] (Figure 5E). These data demonstrate that, similar to XopD^216-760^, XopD^1-760^ displays SUMO protease activity *in planta*.

### Analysis of XopD^1-760^-mediated virulence functions *in planta*

We next investigated whether the newly identified N-terminal protein extension in XopD may have an effect on its function *in planta*. First, a previous report showed that *Agrobacterium*-mediated transient expression of XopD^216-760^ in *N. benthamiana* prevents the induction of the expression of the *PR1* promoter (*PR1p*) fused to the *GUS* reporter gene after salicylic acid (SA) treatment [46]. Consistent with previous results, SA treatment induced *PR1p* transcriptional activation whereas, in the presence of XopD^216-760^, *PR1p* activation was significantly reduced (Figure 6A). Interestingly, co-expression of XopD^1-760^ in these assays led to a stronger repression of *PR1p* transcriptional activation, suggesting that the N-terminal extension of XopD is necessary to modulate XopD function in the host (Figure 6A).

**Figure 6:** *In planta* analysis of XopD^1-760^-mediated virulence functions. (**A**) Transactivation of the *PR1* promoter after SA treatment in transient assays in *N. benthamiana*. Leaves were inoculated with *A. tumefaciens* carrying a *35S:PR1p-GUS* fusion either alone (lanes 1, 2) or together with HA-tagged XopD^216-760^ (lane 3) or XopD^1-760^ (lane 4). 18 hours after agroinfiltration, leaves were mock-treated (white bar) or treated with 2 mM SA (grey bars). Fluorimetric GUS assays in leaf discs were performed 12 hours later. Mean values and SEM values were calculated from the results of four independent experiments, with four replicates per experiment. Statistical differences according to a Student's t test P value <0.05 are indicated by letters. MU, methylumbelliferone. (**B**) Western blot analysis showing expression of HA-tagged XopD^216-760^ and XopD^1-760^. Ponceau S staining illustrates equal loading. (**C**) Susceptible Pearson tomato leaves were inoculated with *Xcv* 85* or *Xcv* 85* Δ*xopD*, expressing an HA-tagged GUS control, *Xcv* 85* Δ*xopD* expressing HA-tagged XopD^216-760^ or *Xcv* 85* Δ*xopD* expressing HA-tagged XopD^1-760^. Inoculation was performed with bacterial suspensions of 1×10^5^ cfu/ml. Representative symptoms observed 10 dpi are shown. Similar phenotypes were observed in four independent experiments. (**D**) Strains *Xcv* 85* expressing a GUS control (1) and 85* Δ*xopD* expressing either a GUS control (2), XopD^216-760^ (3) or XopD^1-760^ (4) were incubated in MOKA rich medium (total extract, left) or secretion medium (supernatant, right). Total protein extracts (10-fold concentrated) and TCA-precipitated filtered supernatants concentrated (200-fold concentrated) were analysed by immunoblotting using anti-HA antibodies (upper panel) to detect the presence of GUS, XopD^216-760^ and XopD^1-760^, or anti-GroEL antibodies (lower panel) to show that bacterial lysis had not occurred.

The article "Detection and Functional Characterization of a 215 Amino Acid N-Terminal Extension in the Xanthomonas Type III Effector XopD" was retracted in 2018. Reasons: manipulated images; duplicated images.

Second, XopD was previously reported to delay the onset of symptom development in susceptible tomato leaves after inoculation with *Xcv* [46]. In order to assess the role of XopD^1-760^ and XopD^216-760^ in *Xcv* symptom development in tomato, we first engineered a XopD null mutant in *Xcv* strain 85*. The sequence encoding the entire XopD ORF (XopD^1-760^) was deleted by homologous recombination to generate an *Xcv* 85* Δ*xopD* mutant strain. In agreement with previously published data, tomato leaves of the susceptible cultivar Pearson inoculated with *Xcv* Δ*xopD* developed cell death by 10 days post inoculation (dpi) whereas leaves inoculated with *Xcv* were relatively healthy at the same time point (Figure 6C). Interestingly, the mutant strain *Xcv* 85* Δ*xopD* expressing wild-type HA-tagged XopD^1-760^ from a constitutive *lac* promoter in a broad host range plasmid was complemented for symptom development, whereas transformation of the same strain with an equivalent construct to express XopD^216-760^ did not allow complementation and inoculated leaves became necrotic (Figure 6C). These data were confirmed by inoculation of susceptible tomato plants of the Moneymaker cultivar, which showed identical results (data not shown). Western blot analysis with an anti-HA antibody showed expression of both XopD^216-760^ and XopD^1-760^ in bacterial total protein extracts (Figure 6D). XopD^216-760^ lacks the first 215 amino acids of XopD, which contain the T3S-dependent secretion signal. As a result, XopD^1-760^, but not XopD^216-760^, could be detected in culture supernatants from bacteria incubated in secretion medium (Figure 6D; lanes 3,4). As expected, the HA-tagged GUS control protein expressed by *Xcv* 85* or *Xcv* 85* Δ*XopD* was detected in total bacterial extracts but not in culture supernatants (Figure 6D; lanes 1,2). These results demonstrate that XopD^1-760^ contains all necessary elements for functional N-terminal secretion and virulence function *in planta*. Together, our data (i) are consistent with XopD being a 760 amino acid protein and (ii) stress the biological significance of the newly identified N-terminal extension of XopD.

The article "Detection and Functional Characterization of a 215 Amino Acid N-Terminal Extension in the Xanthomonas Type III Effector XopD" was retracted in 2018. Reasons: manipulated images; duplicated images.

## Discussion

Prediction of the translation start in bacterial proteins is particularly difficult, rendering systematic annotation of effector proteins a challenging task. Here, we took a mass spectrometry approach to determine the protein sequence of XopD following immunopurification from *Xcv*. After trypsin digestion, 13 peptides were identified upstream the formerly annotated starting M residue, confirming that the XopD protein sequence annotated in the public databases is not complete. Moreover, trypsin digestion of purified XopD led to detection of the peptide IFNFDYK (starting after R^3^ in Figure 3), showing that XopD may start either at the first (UUG codon) or the second (AUG codon) M residue shown in Figures 1C and 3. Detection of the peptide MDRIFNFD, after V8 protease treatment, confirmed that the newly identified N-terminal domain present in XopD produced and secreted by *Xcv* comprises 215 amino acids and that XopD is thus a 760 amino acid protein. This finding is consistent with the observation that initiation of translation of 84% of the predicted *Xcv* ORFs is predicted to start at an AUG codon, whereas only 4% of the predicted *Xcv* ORFs are predicted to start at a UUG triplet. In agreement with this assumption, out of a total of 28 inspected *Xcv* T3Es effectors, none is predicted to be translated starting from a UUG codon. Interestingly, the first predicted UUG codon in XopD from *Xcv* is not present in the XopD coding regions from either *Xcc* B100 or *A. avenae*, whereas the AUG codon, which is used to initiate XopD translation, is well conserved. Finally, inoculation of tomato susceptible plants with *Xcv* expressing XopD^1-760^ provided further confirmation that XopD from *Xcv* is a functional 760 amino acid secreted protein (see below).

In the case of T3Es, the existence of the T3S N-terminal secretion and translocation signals could theoretically help prediction of their starting amino acid. However, secretion signals are not conserved at the amino acid level, even among related or conserved effectors [36], [38] and, in some cases, they are highly tolerant of substitutions [58], [59]. Moreover, in many cases, the presence of several in frame putative initiation codons makes it difficult to determine the starting amino acid for a given effector. Several programs have been developed for prediction of T3S signals in secreted proteins from Gram-negative bacteria [60]–[62]. In the case of XopD, two different recent algorithms [60], [61] assigned the highest probability of secretion to XopD^51-760^, which, as shown in this study, does not correspond to the XopD protein secreted by *Xcv*, whereas the assigned probability of secretion for XopD^1-760^ was very low. This is in agreement with previous reports estimating that algorithm-based gene prediction may lead to up to 40% of wrongly assigned start codons [63]. Indeed, prediction of T3Es secretion is not straightforward, since real translation starts of T3Es have only occasionally been determined experimentally. In a few cases, manual changes of predicted translational start positions have been reported, particularly in the case of myristoylated T3Es, for which the presence of the conserved myristoylation motif facilitates determination of the translation start [64].

The article "Detection and Functional Characterization of a 215 Amino Acid N-Terminal Extension in the Xanthomonas Type III Effector XopD" was retracted in 2018. Reasons: manipulated images; duplicated images.

Several reasons may explain why the newly identified N-terminal extension of XopD was previously overlooked. First, XopD N-terminal extension presents a low coding probability using standard codon usage matrices. Indeed, the G+C content in this genomic region is lower (47%) than in the rest of the *xopD* gene (54%) and much lower than in the rest of the *Xcv* genome (65%), suggesting its acquisition from a different organism with a different codon usage. For instance, the ACUR0 matrix (alternative codon usage regions [65]), developed for systematic annotation of *Ralstonia* T3Es, assigns higher coding probability to this region, although, using this matrix, M^41^ is predicted to be XopD starting amino acid. Indeed, when analyzed for base composition, most ACURs differ significantly from the average 67% G+C content found in the entire genome, with variations ranging from 50–70% G+C content. Furthermore, ACURs are often associated with mobile genetic elements, suggesting that ACURs may have been acquired through horizontal transfer [65]. Interestingly, *xopD* acquisition by horizontal transfer during evolution was previously proposed [47].

T3SS-dependent translocation of XopD into plant cells was previously demonstrated using a translational C-terminal fusion with the calmodulin-dependent adenylate cyclase domain (Cya) of *Bordetella pertussis* cyclocysin [66]. In these assays, 815 bp corresponding to what was previously annotated as the *xopD* promoter region and the annotated XopD coding region (XopD^216-760^) were fused to the CyA sequence and detection of the CyA activity in pepper leaves reflected XopD translocation [43]. However, considering our present findings, the construct used for the CyA assays comprised the N-terminal extension identified here (XopD^1-760^) preceded by a promoter *xopD* region of only 171 bp. Interestingly, this small promoter region appears to contain all necessary elements to allow XopD expression and wrong annotation of XopD was thus not suspected. Likewise, previously reported complementation studies of a *Xcv* strain deleted from XopD were performed with a construct that contained the *xopD* promoter and the complete XopD coding sequence [46]. Although the authors did not describe the length of the *xopD* promoter sequence used for complementation of the *Xcv* Δ*xopD* mutant strain, it must have contained at least the N-terminal extension described in the present work and a promoter region that is long enough to allow complementation.

The article "Detection and Functional Characterization of a 215 Amino Acid N-Terminal Extension in the Xanthomonas Type III Effector XopD" was retracted in 2018. Reasons: manipulated images; duplicated images.

The present study demonstrates that the newly identified N-terminal extension in XopD is essential for its secretion and promotes XopD virulence function(s) *in planta*. First, XopD N-terminal domain appears to negatively regulate XopD-induced cytotoxicity. In addition, XopD^1-760^ is more efficient than XopD^216-760^ in repressing transcription of *PR1* after SA treatment, further confirming the presence of important regulatory elements in the N-terminal stretch of XopD. Finally, inoculation of tomato plants showed that XopD^216-760^ is not secreted from *Xcv* due to the lack of its N-terminal T3S-dependent secretion signal and is thus not able to complement an *Xcv* Δ*xopD* mutant strain. In contrast, XopD^1-760^ is detected in supernatants from bacterial cultures and complements the *Xcv* Δ*xopD* mutant. This observation is consistent with the fact that translation of XopD is initiated at the first AUG codon (XopD^1-760^) and that all necessary elements for functional T3S-dependent secretion and *in planta* translocation are thus present in XopD^1-760^.

XopD was formerly described as a modular protein comprising a DNA-binding domain, two transcriptional repression motifs of the EAR type and a SUMO-protease domain [46]. Here, we describe a previously non-identified protein domain in XopD. Although determining the biological function of this protein domain is clearly beyond the scope of this study, our findings provide intriguing clues to the putative role of XopD N-terminal extension. For example, the fact that XopD KAE-rich domain presents a high probability to form coiled-coil structures, together with gel filtration analysis of XopD^1-760^ expressed in *E. coli*, strongly suggest that the KAE-rich domain is indeed involved in the formation of XopD dimers. Interestingly, detection of XopD dimers was not possible in *Xcv*, perhaps indicating that XopD is unfolded or associated to T3S chaperones prior to its injection in the plant cell. This idea is consistent with previous reports indicating that efficient effector translocation requires the assistance of specialized chaperones that promote the stability and/or secretion of their corresponding interaction partners, keeping them in a partially unfolded and, thus, secretion-competent conformation and guiding them to the secretion apparatus [56], [57]. In protein dimers, cooperativity between the two proteins that form the dimer may increase the binding affinity for DNA [67]. Dimerization can also enhance the specificity of DNA binding by doubling the length of the DNA region bound by the protein dimer [67]. XopD^216-760^ was previously described as a transcriptional repressor of plant target genes that displays non-specific DNA binding activity [46]. Therefore, our finding that the XopD N-terminal extension is involved in dimer formation opens new perspectives regarding the study of XopD specificity of DNA binding as well as the search of its host targets.

The article "Detection and Functional Characterization of a 215 Amino Acid N-Terminal Extension in the Xanthomonas Type III Effector XopD" was retracted in 2018. Reasons: manipulated images; duplicated images.

BLAST analysis of the KAE-rich region with a high propensity to form coiled-coil dimers (residues 177-202; Figure 4A) identified a number of hits corresponding to protein families with a high degree of amino acid sequence homology. Particularly interesting was the homology of this region of XopD with the TolA protein family. TolA are membrane proteins involved in colicin uptake [68]. Interestingly, these proteins also contain a region rich in K, A, E residues that has been shown to form long α-helical structures [69]. The high degree of similarity observed after sequence alignment of this KAE-rich region of TolA with XopD^177-202^ amino acid residues (Figure S3A) suggests that this region of XopD may adopt a similar structural conformation.

Further analysis of the sequence upstream of the KAE-rich region in XopD allowed us to identify a sequence (residues 165–175) with homology to the MarR (Multiple antibiotic resistance) family of proteins (Figure S3B). This family of transcriptional regulators is named after *E. coli* MarR, a repressor of genes that activate multiple antibiotic resistance and oxidative stress regulons [70]. MarR homologs are homodimers that bind sequence-specific palindromic or pseudopalindromic DNA via a winged HTH (helix-turn-helix) motif. The crystal structures of several members of the MarR family show that the winged HTH DNA-binding core is flanked by helices involved in protein dimerization [71], [72]. Interestingly, the XopD sequence containing residues 165–175 shows homology with the DNA recognition helix H3 (α4), which confers specificity of DNA binding to MarR family members [73]. It is noteworthy that XopD^165-175^ sequence, as its homologous sequence in MarR proteins, is located next to a domain (KAE-rich) involved in protein dimerization that may adopt a α-helical structure, based on its homology with the TolA protein family. The DNA recognition helix α4 in MarR proteins contains conserved arginine (R) residues that are also present in XopD (Figure S3B). Mutations in this recognition helix and, in particular, in conserved R73 and R77 residues in *E. coli* MarR, equivalent to R170 and R174 in XopD, abolish MarR DNA binding and repressor activities in whole cells and *in vitro* [73]. More precisely, DNA-binding specificity mediated by the DNA recognition helix α4 in MarR proteins is determined by the specific contact(s) between residue R73 and the operator. Since XopD^216-760^ displays non-specific DNA binding activity [46], it is enticing to suggest that amino acids 165–175 of XopD^1-760^ may confer specificity for DNA recognition. Further studies are required to confirm the putative structural and functional similarities between this region of XopD and *E. coli* MarR proteins. Future work will determine whether this newly identified region in XopD and/or the KAE-rich domain, related to dimer formation, determine the specificity of the DNA binding activity displayed by the XopD protein.

The article "Detection and Functional Characterization of a 215 Amino Acid N-Terminal Extension in the Xanthomonas Type III Effector XopD" was retracted in 2018. Reasons: manipulated images; duplicated images.

Together, our data stress the difficulties associated to correct annotation of T3Es and open new perspectives for future studies on the XopD protein and its virulence-associated functions *in planta*.

## Materials and Methods

### Bacterial strains and plasmids

*Xcv* 85* [54] and 85* Δ*hrcV*, strains carrying the hrpG* mutation which confers constitutive *hrp* gene expression [54] were cultivated overnight at 28°C in MOKA rich medium [74] or in secretion medium (MA) [75]. Plasmids were introduced into *E. coli* by electroporation and into *Xcv* by triparental mating using pRK2073 as helper plasmid [76], [77]. Oligonucleotide primers used for PCR amplification will be provided upon request.

Unless otherwise indicated, plasmids used in this study were constructed by Gateway technology (GW; Invitrogen) following the instructions of the manufacturer. PCR products flanked by the *att*B sites were recombined into the pDONR207 vector (Invitrogen) via a BP reaction to create the corresponding entry clones with *att*L sites. Inserts cloned into the entry clones were subsequently recombined into the destination vectors via an LR reaction to create the expression constructs.

XopD^1-760^ and XopD^216-760^ were amplified from *Xcv* 85-10 genomic DNA. XopD^216-760^ carrying a mutation in the conserved catalytic Cys residue was amplified from a pGEX-XopD^216-760^-C470A vector, kindly provided by Mary Beth Mudgett (Standford University, USA) [43]. 6xHis-, HA-, and YFPv-tagged constructs were generated by recombination of the corresponding entry vectors with pTH19 [78], pBin19-35S-GW-3HA, or pBin19-35S-GW-YFPv destination vectors, respectively (YFPv for YFPvenus, an enhanced form of the YFP; [79]–[80]). For complementation of the *Xcv* 85* Δ*xopD* mutant strain, XopD^1-760^ and XopD^216-760^ were recombined into a pLAFR6-GW-3HA vector (kind gift of Laurent Deslandes, LIPM, Castanet-Tolosan, France) that allows expression of HA-tagged XopD proteins under the control of a constitutive *lac* promoter.

The article "Detection and Functional Characterization of a 215 Amino Acid N-Terminal Extension in the Xanthomonas Type III Effector XopD" was retracted in 2018. Reasons: manipulated images; duplicated images.

For GUS reporter assays in *N. benthamiana*, a 1-kb fragment of the *PR1* promoter (*PR1p*) was amplified from Arabidopsis Col-0 genomic DNA. The PCR product was cloned into the entry vector pDONR207 and subsequently recombined into the pKGWFS7 destination vector [81], resulting in a plant expression vector that contains a transcriptional fusion between the *PR1p* and the *GUS* reporter gene.

### Epitope tagging of XopD and secretion assays

A 307 bp fragment containing the C-terminal end of XopD fused to an HA epitope was amplified by PCR. The amplified fragment was digested with *Bam*HI and *Xba*I and cloned into the suicide plasmid pVO155 [82]. This construct was introduced into the *Xcv* 85* and *Xcv* 85* Δ*hcrV* strains. Secretion experiments were performed as described previously [75] and XopD was detected by Western blot analysis.

### Expression and gel separation of HA-tagged XopD

500 ml of bacteria *Xcv* strain 85* expressing HA-tagged XopD were cultivated overnight at 28°C in MOKA rich medium. The bacterial pellet was washed, resuspended in protein extraction buffer [50 mM Tris-HCl (pH 7.4), 150 mM NaCl, 10% glycerol (v/v), 1 mM DTT, 1 mM PMSF] and lysed using a French Press. Total protein extracts were ultracentrifuged at 100,000 *g* for 30 min at 4°C and the supernatant was subjected to immunoprecipitation using anti-HA affinity matrix (clone 3F10; Roche). Immunoprecipitated proteins were separated on a NuPage 4–12% Bis-Tris gel (Invitrogen) according to the manufacturer's instructions. The proteins were stained using a commercial solution (PageBlue, Fermentas) and the band corresponding to XopD was excised from the gel for subsequent analysis by mass spectrometry.

### Determination of XopD starting amino acid by mass spectrometry

The gel slice containing the XopD protein was digested by incubating with trypsin (Promega, Madison, WI, USA) or V8 protease (Roche) and the resulting peptides were extracted following established protocols [83]. The trypsin digest was then reconstituted in 18 µl 5% acetonitrile, 0.05% trifluoroacetic acid. 5 µL were analysed by nanoLC-MS/MS using an Ultimate 3000 system (Dionex, Amsterdam, The Netherlands) coupled to an LTQ-Orbitrap mass spectrometer (Thermo Fisher Scientific, Bremen, Germany). The peptide mixture was loaded on a C18 precolumn (300 µm ID x 15 cm PepMap C18, Dionex) equilibrated in 95% solvent A (5% acetonitrile, 0.2% formic acid) and 5% solvent B (80% acetonitrile, 0.2% formic acid). Peptides were eluted using a 5 to 50% gradient of solvent B during 80 min at 300 nl/min flow rate. Data were acquired with Xcalibur (LTQ Orbitrap Software version 2.2, Thermo Fisher Scientific). The mass spectrometer was operated in the data-dependent mode and was externally calibrated. Survey MS scans were acquired in the Orbitrap on the 300–2000 m/z range with the resolution set to a value of 60,000 at m/z 400. Up to 5 most intense multiply charged ions (2^+^, 3^+^ or 4^+^) per scan were CID fragmented in the linear ion trap. A dynamic exclusion window was applied within 60 sec. All tandem mass spectra were collected using normalized collision energy of 35%, an isolation window of 4 m/z, and 1 µscan. Other instrumental parameters included maximum injection times and automatic gain control targets of 250 ms and 500,000 ions for the FTMS, and 100 ms and10, 000 ions for LTQ MS/MS, respectively.

The article "Detection and Functional Characterization of a 215 Amino Acid N-Terminal Extension in the Xanthomonas Type III Effector XopD" was retracted in 2018. Reasons: manipulated images; duplicated images.

Data were analyzed using Xcalibur software (version 2.0.6, Thermo Fisher Scientific) and MS/MS centroid peak lists were generated using the extract_msn.exe executable (Thermo Fisher Scientific) integrated into the Mascot Daemon software (Mascot version 2.2.03, Matrix Sciences). Dynamic exclusion was employed within 60 seconds to prevent repetitive selection of the same peptide. The following parameters were set to create peak lists: parent ions in the mass range 400–4,500, no grouping of MS/MS scans, and threshold at 1,000. The data were searched against the protein database of *Xanthomonas campestris pv vesicatoria* 85-10 (NCBI) containing 4411 sequences to which the longest possible ORF for XopD was added (Figure 1C). Mass tolerances in MS and MS/MS were set to 5 ppm and 0.8 Da, respectively, and the instrument setting was specified as “ESI Trap”. Trypsin (specificity set for cleavage after K or R) and V8 (specificity set for cleavage after D or E) were designated as proteases, and one missing cleavage was allowed. Oxidation of methionine was searched as variable modification and carbamidomethylation of cysteine was set as fixed modification. All fragmentation spectra of peptides were manually checked as shown in Figure S1 and S2.

### Protein expression in *N. benthamiana*

*Agrobacterium*-mediated transient expression in *N. benthamiana* leaves was performed as described [84].

The article "Detection and Functional Characterization of a 215 Amino Acid N-Terminal Extension in the Xanthomonas Type III Effector XopD" was retracted in 2018. Reasons: manipulated images; duplicated images.

### Fluorescence Microscopy

YFPv fluorescence in *N. benthamiana* leaves was analyzed with a confocal laser scanning microscope (TCS SP2-SE; Leica) using a x63 water immersion objective lens (numerical aperture 1.20; PL APO). YFP fluorescence was excited with the 514 nm line ray of the argon laser and detected in the range between 520 and 575 nm. Images were acquired in the sequential mode (20 Z plains per stack of images; 0.5 µm per Z plain) using Leica LCS software (version 2.61).

### XopD expression in *E. coli*

Expression vectors containing 6xHis-tagged XopD^1-760^ and XopD^216-760^ were transformed in *E. coli* Rosetta cells. For expression of recombinant proteins, cells were grown in Luria-Bertani (LB) medium at 28°C to OD_600_  = 0.6 to 0.8 and then induced with 0.2 mM isopropylthio-β-galactoside (Roche) for 4 h at 28°C. Cells were lysed in PBS, pH 8.0 and 1 mM phenylmethylsulfonyl fluoride (Sigma-Aldrich) using a French Press.

### Gel Filtration Analysis

Gel filtration was performed using a fast protein liquid chromatography system (Pharmacia) with HR 10/30 Superdex S-200 high-resolution columns (Pharmacia). Prior to chromatography, protein extracts were ultracentrifuged to remove any aggregates. All gel filtration assays were performed at 4°C with pre-filtered protein extracts. Column equilibration and chromatography were performed in PBS buffer. Fractions were collected every 0.4 ml and analyzed by Western blot.

### Protein Gel Blot Analysis

Proteins were separated on NuPage 4%–12% Bis-Tris gels (Invitrogen) following the manufacturer's instructions and transferred onto Protran BA85 nitrocellulose membranes (Schleicher & Schuell) by wet electroblotting (Mini-Protean II system; Bio-Rad). For detection of HA-, YFPv- and His-tagged proteins, blots were respectively incubated with rat monoclonal anti-HA [clone EF10 (Roche); 1∶5,000] and mouse monoclonal anti-His6-peroxidase [clone-His-2 (Roche); 1∶50,000] antibodies, linked to horseradish peroxidase. Anti-GroEL rabbit polyclonal (Stressgen Biotechnologies Corporation) and mouse monoclonal anti-GFP IgG1 K [clones 7.1 and13.1 (Roche)] were used at 1∶10,000. Proteins were visualized using the Immobilon kit (Millipore) under standard conditions.

### Fluorimetric GUS Assays

For GUS reporter assays, the indicated constructs were transiently expressed in *N. benthamiana* leaves using *Agrobacterium*. Leaves were sprayed with 2 mM salicylic acid (SA; SIGMA-Aldritch) 18 hours after agroinfiltration. 12 hours later, leaf discs were collected, frozen in liquid nitrogen and stored at −80°C until processing. GUS activity was measured using the substrate 4-methylumbelliferyl-β-D-glucuronide as described previously [80]. After protein extraction, 1 µg of total protein was used in replicates to measure enzymatic GUS activity of individual samples.

The article "Detection and Functional Characterization of a 215 Amino Acid N-Terminal Extension in the Xanthomonas Type III Effector XopD" was retracted in 2018. Reasons: manipulated images; duplicated images.

### Construction of a *Xcv* 85* Δ*xopD* deletion mutant strain

An *Xcv* 85* *xopD* deletion mutant strain was constructed by using the *sacB* system [85]. Briefly, 830 bp upstream and 850 bp downstream regions of full-length *xopD* were amplified by PCR using *Xcv* 85-10 gDNA as template. PCR products were subsequently cloned in a GoldenGate-compatible pK18 plasmid (L. Noël, unpublished). GoldenGate is a cloning method based on the use of Type II restriction enzymes, *Bsa*I in our study [86]. This plasmid was then introduced into *Xcv* 85* by triparental mating and deletion of *xopD* was verified by PCR.

For complementation of the *Xcv* 85* Δ*xopD* mutant strain, pLAFR6 vectors carrying either an HA-tagged GUS control (kind gift of Laurent Deslandes, LIPM, Castanet-Tolosan, France), XopD^216-760^ or XopD^1-760^ were introduced into *Xcv* 85* Δ*xopD* by triparental mating.

### Inoculation of susceptible tomato cultivars

Whole leaves of *Solanum lycopersicum* cv Moneymaker or cv Pearson were inoculated with a 1×10^5^ cfu/mL suspension of bacteria in 10 mM MgCl_2_ using a needleless syringe. Leaves of the same age on the same branch were used for each experimental test. Plants were kept under 16 h light/day at 28°C. Symptoms were analyzed 10 days after plant inoculation.

### Quantification of cell death using electrolyte leakage

For electrolyte leakage measurements, 8 *N. benthamiana* leaf discs (6 mm diameter) were harvested 24 hours after agroinfiltration, washed and incubated at room temperature in 10 ml of distilled water before measuring conductivity.

## Supporting Information

Figure S1 **MS/MS spectra of peptides issued from tryptic hydrolysis of the XopD protein.** Peptides were analyzed by LC-MS/MS using a capillary LC system coupled directly to an LTQ-Orbitrap mass spectrometer. Each MS/MS spectrum is a collection of ions produced by collision-induced dissociation of the intact peptide in the linear ion trap. The predominant b and y product ion peaks are labeled accordingly with the subscripts denoting their position in the identified peptide and 2^+^ or 3^+^ indicating doubly or triply protonated ions respectively. y and b ions that were detected on the graph are shown in bold.
(DOC)

Figure S2 **MS/MS spectra of peptides issued from V8 hydrolysis of the XopD protein.** Peptides were analyzed by LC-MS/MS using a capillary LC system coupled directly to an LTQ-Orbitrap mass spectrometer. Each MS/MS spectrum is a collection of ions produced by collision-induced dissociation of the intact peptide in the linear ion trap. The predominant b and y product ion peaks are labeled accordingly with the subscripts denoting their position in the identified peptide and 2^+^ or 3^+^ indicating doubly or triply protonated ions respectively. y and b ions that were detected on the graph are shown in bold.
(DOC)

Figure S3 **Bioinformatics analysis of the N-terminal region of XopD.** (**A**) Alignment of amino acid residues 177-202 of XopD with its homologous regions of the following proteins from the TolA family: TolA from *Aeromonas salmonicida* (A4SJ34), *Erwinia chrysantemi* (Q937K4), *Escherichia coli* (P19934), *Haemophilus influenzae* (P44678), *Pseudomonas aeruginosa* (P50600), *Salmonella typhi* (Q8Z8C1), *Shewanella oneidensis* (Q8EDJ7), *Shigella dysenteriae* (Q32II2), *Tolumonas auensis* (C4LBM3), *Vibrio harveyi* (A6AM98). (**B**) Alignment of amino acid residues 168-177 of XopD with its homologous regions of the following proteins from the MarR family: MarR from *Escherichia coli* (P27245), *Enterobacter cloacae* (Q9F4W7), *Salmonella typhimurium* (P0A2T4), *Shigella flexneri* (Q0T4J9), *Citrobacter youngae* (D4B9P6), *Tolumonas auensis* (C4LFI7), *Bordetella petrii* (A9ITE7), *Burkholderia pseudomallei* (Q63Z16), *Klebsiella pneumoniae* (C8T9Z4), *Pseudomonas aeruginosa* (B7V3Q1), *Pseudomonas fluorescens* (Q4K9R4), *Pseudomonas putida* (BIJ789), *Pseudomonas syringae* (Q48FY2). Positions of the conserved Arg residues responsible for DNA binding in MarR family members are indicated by an asterisk. Percentage of sequence identity is represented by colour intensity of blue boxes.
(DOC)
